# The Emerging Role of Noncoding RNA Regulation of the Ferroptosis in Cardiovascular Diseases

**DOI:** 10.1155/2022/3595745

**Published:** 2022-09-21

**Authors:** Jing Zhang, Xinran Liu, Xiaozhong Li, Yuxi Cai, Yiwen Zhou, Qiong Wang, Zhou Xu, Panpan Xia, Pingping Yang, Lei Jun, Peng Yu, Ao Shi

**Affiliations:** ^1^Department of Anesthesiology, The Second Affiliated Hospital of Nanchang University, Jiangxi, Nanchang 330006, China; ^2^Queen Mary College of Nanchang University, Nanchang, China; ^3^Department of Cardiology, The Second Affiliated Hospital of Nanchang University, Jiangxi, Nanchang 330006, China; ^4^The Second Clinical Medical College of Nanchang University, The Second Affiliated Hospital of Nanchang University, Jiangxi, Nanchang 330036, China; ^5^Medical College of Tibet University, Lhasa, Tibet Autonomous Region 850000, China; ^6^Department of Endocrinology and Metabolism, The Second Affiliated Hospital of Nanchang University, Jiangxi, Nanchang 330006, China; ^7^Department of General Surgery, The Second Affiliated Hospital of Nanchang University, Jiangxi, Nanchang 330006, China; ^8^St. George's, University of London, London, UK; ^9^School of Medicine, University of Nicosia, Nicosia, Cyprus

## Abstract

Cardiovascular disease (CVD) is a significant public health issue due to its high prevalence and considerable contribution to the global disease burden. Recent studies suggest that genetic factors, including noncoding RNAs, have an important role in the progression of CVD. Noncoding RNA plays a critical role in genetic programming and gene regulation during development. Ferroptosis is a form of iron-dependent regulated cell death (RCD), which is mainly caused by increased lipid hydroperoxide and redox imbalance. Ferroptosis is essentially different from other forms of RCD in morphology and mechanism, such as apoptosis, autophagic cell death, pyroptosis, and necroptosis. Much evidence suggested ferroptosis is involved in the development of various CVDs, especially in cardiac ischemia/reperfusion injury, heart failure, and aortic dissection. Here, we review the latest findings based on noncoding RNA regulation of ferroptosis and its involvement in the pathogenesis of CVD and related treatments, aimed at providing insights into the impact of noncoding RNA regulation of ferroptosis for CVD.

## 1. Introduction

Ferroptosis is a nonapoptotic form of cell death, which is attributed to abnormal cellular iron levels that lead to increased accumulation of lipid peroxides [1]. From this perspective, ferroptosis is also an iron-dependent form of regulated cell death (RCD). Compared with other forms of cell death, ferroptosis has its unique characteristics in morphology, biochemistry, and genetics. The ferroptosis cell includes dense and compact mitochondria without cristae and loss of plasma membrane integrity. Ferroptosis induced by erastin and Ras selective lethal small molecule 3 (RSL3) is inhibited via iron chelators [2]. At present, a large number of studies have shown that the regulation mechanism of ferroptosis involves multiple signaling and metabolic pathways, especially the glutathione peroxidase 4 (GPX4) axis. In particular, by inhibiting the system x_c_^−^, the GPX4 axis x_c_^−^ leads to decreased cysteine levels and glutathione (GSH) deficiency, contributing to excessive accumulation of lipid peroxides [3–5]. Current studies have shown that ferroptosis has an important impact on many diseases, such as neurodegenerative diseases, cardiovascular disease, cancer, and ischemia-reperfusion injury [6–9].

Noncoding RNA (ncRNA) is the RNA molecules transcribed from genomes that do not encode proteins. ncRNA is not only important to transcriptional and posttranscriptional levels but also plays a significant role in epigenetic regulation of gene expression. Recent studies have revealed that about 90% of the genes in eukaryotic genomes are transcriptional genes. Interestingly, only 1-2% of these transcribed genes encode proteins. Most genes are transcribed as ncRNAs.

There are two subtypes of ncRNA, including basic structural and regulatory ncRNA. The former plays a role as a housekeeping gene during the translation and splicing, which includes ribosomal RNA, transfer RNA, and small nuclear RNA. From an epigenetic point of view, regulatory ncRNA matters more, because it involves the modification of other RNA. The regulatory ncRNA contains microRNA (miRNA), piwi-interacting RNA (piRNA), small interfering RNA (siRNA), and long noncoding RNA (lncRNA). At present, a large number of studies have demonstrated ncRNAs as cardinal regulators to regulate a series of genetic process including transcription and translation [10–12].

With the in-depth research, a large number of human diseases have been considered to correlate with gene expression under the regulation of ncRNA [13], including cancer, viral infection, neurodegenerative diseases, and cardiovascular diseases [14–18]. From this aspect, an overall understanding of the biological function and mechanism of ncRNA will help to better understand the molecular basis of the disease and develop new therapeutic strategies.

Here, we conducted a comprehensive review on whether ncRNAs affect ferroptosis in cardiovascular disease and critically analyzed the mechanism of action between ncRNAs and ferroptosis in cardiovascular diseases. We aim to (i) provide insights into the ncRNA-regulated ferroptosis, (ii) emphasize that ncRNAs are involved in the regulation of ferroptosis in cardiovascular diseases, and (iii) explore the possibility of using ncRNAs as targets to interfere with ferroptosis in cardiovascular diseases.

## 2. Ferroptosis and Iron Metabolism in Cardiovascular Diseases

At present, studies have revealed that programmed cell apoptosis is closely related to the occurrence and development of cardiovascular disease [19]. Dixon et al. first proposed the concept of ferroptosis in 2012. Ferroptosis is a nonapoptotic form of cell death, which differs from the morphological, biochemical, and genetic manifestations of apoptosis, necrosis, and autophagy [1]. Research has described the mechanism of central nerve cell ferroptosis and found that the mechanism is different compared to apoptosis. Earlier, this type of cell death was called ‘oxidative glutamate toxicity' or ‘oxytosis' [20]. Further studies have manifested that ferroptosis is related to iron overload, free polyunsaturated fatty acid (PUFA) oxidation, and redox pathway impairment [21, 22].

The iron metabolism pathway is the key to ferroptosis. Fe^2+^ reacts with ceruloplasmin to convert to Fe^3+^, which then binds to transferrin (TF) to form a complex. The complex is endocytosed into cells by membrane protein TF receptor 1 (TFR1) [23, 24]. Intracellular Fe^3+^ is stored in unstable iron pools (LIP) and ferritin is reduced to Fe^2+^ for the synthesis of iron-dependent enzymes [25, 26] and increased iron input from iron transporter 1 (FPN1), poly copper-iron oxidase (e.g., ceruloplasmin) and ion transporter lipocalin 2 (LCN2). Eventually, the cells become overloaded with iron [24–28]. Unstable iron pools, especially ferrous iron-induced Fenton reaction, produce a large number of lipid-free radicals triggering ferroptosis.

Glutathione (GSH) and system x_c_^−^ play an important role in iron death. GSH is one of the key reductants in vivo and enables to maintain the redox state of cells. System x_c_^−^, as a cystine-glutamate exchanger, is composed of two proteins, including 12 channel transmembrane protein transporter solute vector family 7 member 11 (SLC7A11) and single-channel transmembrane regulatory protein solute vector family 3 members 2 (SLC3A2). Cystine and glutamate are exchanged in equal proportions by the system x_c_^−^. GSH is synthesized by cysteine, glutamate, and glycine in two steps.

With GSH, GPX4 eliminates lipid peroxides by reducing the presence of complex phospholipid hydroperoxides (PL-OOH) in cell membranes, thus preventing ferroptosis [29, 30]. The specific mechanism of ferroptosis is illustrated in Figure 1.

Recently, many studies have indicated that ferroptosis also has an important effect on cardiovascular disease. Fang et al. found that the mechanism of doxorubicin (DOX) induced cardiomyopathy by upregulating heme oxygenase-1 (Hmox1) through Nrf2, which degrades heme, increases free iron in cardiomyocytes, leads to lipid oxidation, and then damages mitochondrial structure and function [31]. This study also showed that the ferroptosis inhibitor, ferrostatin-1 (Fer-1), and the iron chelator, dexrazoxane (DXZ), alleviate DOX-induced cardiomyopathy by improving mitochondrial function and mitochondrially targeted antioxidant (MitoTEMPO) by reducing lipid overload oxidation inhibits ferroptosis, thereby reducing DOX-induced cardiomyopathy [31]. Studies have shown that Fer-1 can relieve diabetic myocardial ischemia-reperfusion injury (IRI), since Fer-1 inhibits ferroptosis by improving endoplasmic reticulum stress and reducing reactive oxygen species (ROS) levels [32]. After cardiac ischemia-reperfusion (IR), the cardiomyocytes around the scar tissue appear iron deposition. The increase of intracellular iron level induced lipid oxidation, thus leading to ferroptosis, while mTOR restrained ferroptosis by affecting the iron metabolism of cardiomyocytes [33]. Similarly, liproxitatin-1 (Lip-1) protects the myocardium from IRI by increasing the activity of GPX4 to inhibit lipid peroxidation, reducing ROS levels and maintaining the integrity of mitochondrial, thereby inhibiting ferroptosis [34]. Moreover, puerarin treatment improves heart failure by inhibiting NOX4 activity, inhibiting iron droop, and maintaining the integrity of the mitochondrial structure [35]. Lipid oxidation induced by lipopolysaccharide (LPS) leads to ferroptosis and myocardial damage. Therefore, myocardial damage was significantly improved after using Fer-1 [36].

## 3. Noncoding RNA in Ferroptosis Regulation

### 3.1. Noncoding RNA

Most human RNA transcripts do not encode proteins, so they are called ncRNAs, which were used to be regarded as “junk” DNA [37]. In the ENCODE project in 2012, researchers conducted an in-depth study of the so-called “junk” DNA and found that at least 80% of the human genome is biologically functional [37]. They play an important role as *cis*-/*trans*-regulatory elements, introns, pseudogenes, repetitive sequences, and telomeres. At present, ncRNA is mainly classified according to its length and function. In terms of length, it is divided into small RNA (18-200 nt) and long ncRNA (>200 nt); small RNA includes ribosomal RNA (rRNA), transfer RNA (tRNA), microRNA (miRNA), and piwi-interacting RNA (piRNA). Functionally, they are divided into housekeeping ncRNAs such as rRNA and tRNA, and regulatory transcripts such as miRNA, long noncoding RNA (lncRNAs), and circular RNA (circRNA). It is found that ncRNA plays a functional role in remote tissues, which also means that ncRNA plays a part in a variety of biological functions through various mechanisms. miRNA is essential in the regulation of human diseases, especially in cancer progression [10, 13]. When miRNA is overexpressed or inhibited, it activates a complex network of molecular signals and leads to carcinogenesis [38]. The functions of lncRNA and miRNA are similar. lncRNA regulates gene expression such as protein translation and posttranscriptional silencing. Besides, lncRNA represses the translation of *cis*- and *trans*-genes through histone adornment or destroys the miRNA regulation [39, 40]. With different structures from linear messenger RNA (mRNA), there are many types of circRNA with complex functions which include the occurrence and development of diseases. For example, ncRNA is involved in the progression of diabetes and other diseases [13, 41].

### 3.2. The Direct Function of Noncoding RNA

Some ncRNA can target the mRNA directly and regulate relevant proteins, including GSH, ferroportin, and mitoferrin. Ding et al. found that miR-182-5p and miR-378a-3p negatively regulate the expression of GPX4 and SLC7A11 by directly binding the 3′UTR (untranslated region) of GPX4 and SLC7A11 mRNA to promote ferroptosis [42]. In the preeclampsia model, miR-30b-5p downregulates Cys2/glutamate antiporter and PAX3 and reduces the expression of ferroportin 1 (ferroportin), resulting in decreased GSH and unstable Fe2^+^, thereby enhancing ferroptosis [43]. In radiation-resistant cells, miR-7-5P inhibits iron droop by inhibiting the expression of mitoferrin and thereby reducing the iron level [44]. In addition, miR-9 and miR-137 enhance ferroptosis by reducing intracellular GSH levels. Respectively, miR-9 inhibits the synthesis of GSH, while miR-137 inhibits solute carrier family 1 member 5 (SLC1A5), which is a component of system x_c_^−^31 [45]. miR-541-3p inhibits GPX4 axis activity and induces ferroptosis. In ovarian cancer, miR-424-5p negatively regulates ferroptosis by directly targeting ACSL4 in ovarian cancer cells. The upregulation of miR-424-5p inhibits ACSL4 by directly binding 3′UTR, thereby reducing the ferroptosis induced by erastin and RSL3 [46].

### 3.3. The Indirect Function of Noncoding RNA

On the other hand, some ncRNA induced methylation modification and posttranscriptional regulation of related protein, or promote ferroptosis indirectly via the activation of the upstream protein. Zhang et al. found that miR-522 inhibits ferroptosis in gastric cancer by inhibiting the activity of arachidonic acid lipoxygenase 15 (ALOX15) [47]. Clinical evidence shows that ALOX15 is closely related to the production of lipid ROS in gastric cancer. When miR-522 acts on ALOX15, the activity of ALOX15 is inhibited and reduces the accumulation of lipid ROS in cancer cells, thus improving the ferroptosis of gastric cancer cells. Most importantly, they found that ubiquitin-specific protease 7 (USP7) stabilizes heterogeneous ribonucleoprotein A1 (hnRNPA1) through deubiquitination, and hnRNPA1 mediates the filling of miR522 into exosomes. In addition, cisplatin and paclitaxel promote the secretion of miR-522 by cancer-associated fibroblasts via activating the USP7/hnRNPA1 axis. This leads to ALOX15 inhibition and a decrease in the level of lipid ROS in cancer cells, which is also related to the acquisition of drug resistance in gastric cancer. Wang et al. showed that lncRNA-LINC00618 can also induce ferroptosis in leukemia cells by inhibiting the expression of lymphoid-specific helicase (LSH) [48]. LSH was recruited to the promoter region of SLC7A11 and inhibited the expression of SLC7A11, then activating ferroptosis. On the other hand, p53 induces apoptosis or ferroptosis by reducing the accumulation of ROS [49, 50]. Studies have indicated that LNCRNAP53RRA binds to Ras GTP activator protein-SH3 domain binding protein 1 (G3BP1) and replaces p53 in the G3BP1 complex leading to a higher retention rate of p53 in the nucleus and downgrading SLC7A11140, which caused to apoptosis and ferroptosis [51]. LINC00336 is promoted by lymphoid-specific helicase in lung cancer and inhibits iron droop through sponging miR-685232 [52]. In gliomas, circ-TTBK2 has been activated by cavernous miR-761 and subsequent ITGB8 and inhibited IRC-TTBK2 to promote derastin-induced ferroptosis [53].

## 4. Regulation of Noncoding RNA on Ferroptosis in CVD

### 4.1. miRNAs and Ferroptosis in CVD

miRNA is an endogenous noncoding single-stranded small RNA molecule, which is composed of 21-23 bases. The role of miRNAs is to hybridize with part of the UTR of mRNA, causing mRNA to be cleaved or inhibiting mRNA translation. Research has demonstrated that a miRNA can regulate different target genes. Besides, several different miRNAs can jointly regulate a target gene [54].

miRNAs play an important regulatory role in the pathophysiology of CVD [55]. Recently, related studies have been conducted on whether miRNAs affect ferroptosis in CVD. Studies have shown that miR-17-92 inhibits endothelial cell ferroptosis by targeting the A20-ACSL4 axis. The miR-17-92 cluster can mediate angiogenesis, maintain vascular integrity, and protect endothelial cells from ferroptosis induced by oxidative stress [56]. Zhou et al. indicated that miR-190a-5p has an important role in regulating cardiomyocyte ferroptosis. miR-190a-5p negatively regulates ferroptosis by inhibiting GLS2 expression in rat cardiomyocytes. Overexpression of miR-190a-5p will inhibit GLS2 and decrease the accumulation of ROS, MDA, and Fe. At the same time, inhibiting the expression of miR-190a-5p leads to the upregulation of GLS2, which increases the oxidative stress response and ferroptosis [57]. Moreover, Sun et al. found that miR-135b-3p promotes ferroptosis by targeting GPX4, thereby aggravating myocardial ischemia/reperfusion injury. The specific mechanism is as follows: miR-135b-3p downregulates the expression of GPX4, leading to ferroptosis in cardiomyocytes and aggravating myocardial ischemia/reperfusion injury, which means that miR-135b-3p promotes cell death in an iron-dependent manner *in vitro* [58]. Studies have found that knocking out miR-15a-5p can reduce the cell mortality of hypoxic-treated cardiomyocytes, and GPX4 is the direct target of miR-15a-5p. Overexpression of miR-15a-5p enhances iron death, which in turn aggravates the hypoxia damage of cardiomyocytes [59]. At the same time, Song et al. showed that the level of miR-143-3p in atrial fibrillation cardiomyocytes is lower than that in normal cells. Therefore, when miR-143-3p is highly expressed, it can inhibit oxidative damage. And cell ferroptosis mediated by glutamate-oxaloacetate aminotransferase 1 activity can improve the viability of cardiomyocytes and promote proliferation [60]. Additionally, Tang et al. found that miR-30d inhibits autophagy through ATG5 binding, upregulates the expression of FTH1 and GPX4 in H9C2 cells, inhibits ferroptosis of H9C2 cells, and protects myocardial I/R injury [61]. Similarly, miR-29b-3p can also aggravate cardiomyocyte I/R injury by downregulating the expression of PTX3 to exacerbate the inflammatory response [62]. Also, miRNA has an important effect on the prognosis of heart failure. Wang et al. showed that miR-351 overexpression can improve heart failure by inhibiting the expression of MLK3. The specific mechanism is that miR-351 targets MLK3 and inhibits the oxidation mediated by the N JNK/p53 signaling pathway. Finally, stress and ferroptosis lead to myocardial fibrosis in the advanced stage of chronic heart failure [63].

### 4.2. lncRNA and Ferroptosis in CVD

Long noncoding RNAs (lncRNAs) are transcripts that are longer than 200 nucleotides but do not encode protein [64]. lncRNAs control gene expression through *cis*- or *trans*-regulation of chromosome structure, transcription, splicing, mRNA transport, stability, and translation, thus extensively affecting many cellular processes. At present, studies have shown that lncRNAs play a vital role in biological functions [65]. For example, Wang et al. identified that the lncRNA of HAND2-AS1 is highly expressed in liver cancer cells. HAND2-AS1 can make liver cancer stem cells self-renew and promote liver cancer [66]. Previous studies have shown that lncRNA may have an important impact on the occurrence of diabetes. Akerman et al. found that lncRNA is involved in the regulation of *β* cell-specific transcription factor network. PLUTO of a lncRNA encodes a key *β* cell transcription factor by affecting chromatin structure and PDX1 transcription. It was also found that the levels of PLUTO and PDX1 were decreased in the islets of donors with type 2 diabetes or impaired glucose tolerance [67].

Recently, studies have found that lncRNAs can be used as biomarkers for many cardiovascular diseases. Ye et al. indicated that the myocardial infarction-associated transcript (MIAT)/miR-149-5p/CD47 pathway of macrophages plays an important role in the formation of atherosclerotic plaques. The decrease in MIAT level can alleviate the progression of atherosclerosis, stabilize plaque, and promote the clearance of apoptotic cells by macrophages. MIAT is a tiny ribonucleic acid sponge and regulates the expression of the antiphagocytic molecule CD47 through the sponge miR-149-5p [68]. Studies have shown that lncRNA-p21 inhibits cell proliferation and neointima formation in damaged carotid arteries. MDM2 interacts with lincRNA-p21 to promote the expression level of p53 [69]. Klattenhoff et al. thought that lncRNA has a key role in mammalian cardiovascular development. They attested that Braveheart (Bvht) is a heart-related lncRNA and found that Bvht is necessary for the development of the neonatal mesoderm to the fate of the heart. Moreover, Bvht acts upstream of MesP1 (post-mesoderm 1), which is the main regulator of common pluripotent cardiovascular progenitor cells. Bvht also interacts with SUZ12, a component of polycomb inhibitory complex 2 (PRC2), indicating that Bvht can regulate epigenetics in the heart [70]. Wang et al. found that lncRNA-XXYLT1-AS2 is less distributed in atherosclerotic plaques. XXYLT1-AS2 promotes FUS expression and reduces CCND1 expression, thereby blocking the proliferation and migration of human umbilical vein endothelial cells. At the same time, the silencing of XXYLT1AS2 promoted the activation of NF-*κ*B and AKT signals, leading to increased expression of adhesion molecules [71]. Sun et al. showed that lncRNA-UCA1 exerts a cardioprotective effect through the miR-873-5p/XIAP axis under hypoxia. The plasma levels in patients with acute myocardial infarction containing exosomes rich in lncRNA-UCA1 are significantly higher than those in normal populations. Further studies have found that lncRNA-UCA1 targets miR-873 through sponge action, upregulating XIAP expression, thereby promoting AMPK phosphorylation and antiapoptosis [72].

Wang et al. showed that lncRNA-LINC00336 as an oncogene promotes tumor cell proliferation, inhibits ferroptosis, and induces tumorigenesis in an ELAV1-dependent manner [73]. Studies have indicated that lncRNA PVT1 regulates ferroptosis through miR-214-mediated TFR1 and TP53 expressions. Specifically, PVT1 silencing or miR-214 overexpression significantly reduces infarct size and inhibits ferroptosis in vivo [74]. Also, Yang et al. demonstrated the role of the lncRNA ZFAS1/miR-150-5p/SLC38A1 axis in the progression of pulmonary fibrosis. lncRNA ZFAS1 acts as a competitive endogenous RNA (ceRNA) and sponge miR-150-5p to downregulate the expression of SLC38A1 to attenuate iron death and the progression of pulmonary fibrosis [75]. Ni et al. found that lncRNA-ZFAS1 as a ceRNA sponge miR-150-5p can regulate CCND2, thereby promoting ferroptosis in diabetic cardiomyopathy (DCM). Inhibiting lncRNA-ZFAS1 leads to decreased collagen deposition, decreased cardiomyocyte apoptosis and ferroptosis, and the progress of DCM weakened [76]. DOX promotes the activity of lncRNA KCNQ1OT1 by upregulating the expression of METL14, thereby inhibiting the activity of miR-7-5p, increasing the level of transferrin receptor, promoting iron absorption and the production of lipid reactive oxygen species, and inducing cardiomyocyte ferroptosis [77].

### 4.3. circRNA and Ferroptosis in CVD

In back splicing, the downstream (3′) splice donor site reversely accesses the upstream (5′) splice acceptor site, resulting in the formation of covalently linked circRNAs, lack of 5′ caps and 3′ poly-A tails. This makes circRNAs resistant to exonuclease RNase R digestion, so circRNAs are more stable than linear ribonucleic acid. Initially, circRNAs were considered waste products from abnormal splicing events. Only testis-specific circular ribonucleic acid of the sex determining region Y (Sry) gene may be functional [78]. In recent years, with the development of high-throughput sequencing technologies, researchers have found that circRNAs are widely expressed in eukaryotes. At present, it is reported that circRNAs have been related to various human diseases. Studies have found that compared with the normal population, for the patients with type 2 diabetes, the level of circANKRD36 is significantly upregulated. It is related to chronic inflammation of type 2 diabetes [79]. circRNA is generally upregulated during neuronal differentiation, especially highly enriched in synapses, and is negatively correlated with the expression of RNA editing enzyme ADAR1. Therefore, knocking down ADAR1 will increase the expression of circRNA [80]. The proliferation and invasion of rectal cancer cells were inhibited by the new protein circPLCE1-411 encoded by the circular RNA circPLCE1. Dissociated RPS3 from the complex inhibits nuclear translocation of NF-*κ*B in colorectal cancer cells [81]. Holdt et al. indicated that the circular antisense noncoding RNA in circANRIL slows down the development of atherosclerosis by regulating the maturation of rRNA and affecting the formation of atherosclerosis, thus attenuating the development of atherosclerosis [82].

With the continuous deepening of circRNA and ferroptosis research, whether circRNA can impact CVD by regulating ferroptosis has become a focus of attention. Li et al. found that circRNA1615 is inhibited ferroptosis by miRNA152-3p/LRP6 axis regulated cell autophagy in cardiomyocytes of myocardial infarction. Moreover, a previous study showed that Ferrostatin-1, a ferroptosis inhibitor, has an important function in protecting myocardial infarction and reperfusion injury via suppressing ferroptosis [33]. LRP6 has a significant effect on the process of ferroptosis. circRNA1615 regulated the expression of LRP6 through sponge adsorption of miR-152-3p. Then, it prevents ferroptosis mediated by autophagy in cardiomyocytes [83]. Zheng et al. showed that low expression of circSnx12 and high expression of miR-224-5p can downregulate the expression of FTH1 to make myocardial cells iron overloaded, thus leading to ferroptosis. The specific mechanism is that circSnx12 promotes the expression of FTH1 via inhibiting the expression of miR-224-5p, then maintaining an iron steady state in the cell [84].  Table 1 shows the mechanism of noncoding RNAs regulating ferroptosis in CVD.

## 5. Potential Drugs Targeting Noncoding RNA-Regulated Ferroptosis in CVD

Endothelial cell death is associated with vascular diseases such as arteriosclerosis and tissue ischemia. Erastin was utilized by Hong et al. to trigger ferroptosis in HUVEC cells. They discovered that miR-17–92 protects HUVEC cells against ferroptosis by inhibiting the A20-ACSL4 axis [85]. Wu et al. confirmed that miR155-5p inhibits ACE mRNA and protein expression, as well as superoxide anion generation, NAD(P)H oxidase (NOX) activity, NOX2, interleukin-1 (IL-1), and tumor necrosis factor (TNF) expression levels in vascular smooth muscle cells (VSMC). However, miR155-5p did not influence VSMC migration produced by exogenous Ang II [86]. What is more, a recent study shows that miR-15a-5p inhibits Bcl-2 expression in cardiomyocytes to protect the myocardium from apoptotic damage during cardiac surgery [87]. In Xu et al.'s study, Icariside II can target miR-7-5p to suppress the expression of BTG2, thus protecting H9c2 cells from myocardial infarction by upregulating miR-7-5p. Similarly, miR-7 is a downstream factor of curcumin and can be upregulated by curcumin. At the same time, this pathway can also downregulate the expression of the RelA p65 protein to inhibit cellular inflammation and oxidative stress in I/R injury [88].

The related mechanism of of drugs treating CVD is shown in Table 2.

## 6. Conclusions

In recent years, research on non-coding RNA and ferroptosis has continued to progress. A large number of studies have shown that both are involved in the occurrence and development of a variety of cardiovascular diseases. Noncoding RNA is widely expressed in the cardiovascular system and plays an important role in the occurrence and development of cardiovascular diseases (98). Specially, ncRNA crosslinked ferroptosis and CVDs. Ferroptosis is triggered by lipid oxidative stress and iron excess, and ncRNAs can regulate the expression of genes associated with different ferroptosis-related events, including iron homeostasis (FTH1) [84], cell protection (miR-17-92) [56], iron importation (CicSnx12) [83], and oxidative-stress attenuation (miR-143-3p) [60]. However, whether noncoding RNA regulates ferroptosis and thus affects the pathophysiology of cardiovascular diseases remains to be further studied. At present, many studies are confirming that miRNAs participate in the process of cardiovascular disease by regulating ferroptosis. However, there are not many studies on lncRNA and circRNA in this area, understanding their mechanisms and designing effective therapies are urgently needed.

## Figures and Tables

**Figure 1:** Iron metabolism, system x_c_^−^, and lipid peroxides accumulation in ferroptosis. By using TFR1-mediated endocytosis, transferrin transfers iron into cells. Through the Fenton reaction and lipid oxidation, Fe2+ can thereby encourage the formation of lipid peroxides. By importing cysteine, the cofactor of GPX4 allows system xc^−^ to remove lipid peroxides. Ferroptosis may be triggered by an excess of free iron and decreased GPX4 activity.

**Table 1:** Noncoding RNAs regulating ferroptosis in CVD.

ncRNA and expression	Target and expression	Mechanism	Phenomenon	Diseases	Reference
miRNA-17-92 ↑	A20 ↓	Inhibits A20-ACSL4 axis	The proliferation of HUVEC cells	Atherosclerosis disease	[56]
miR-135b-3p ↑	Gpx4 ↓	Inhibits Gpx4 pathway	Promotes the myocardial I/R injury	Myocardial I/R injury	[58]
miR-15a-5p ↑	Gpx4 ↓	Inhibits Gpx4 pathway	Promotes the myocardial I/R injury	Myocardial I/R injury	[59]
miR-29b-3p ↑	PTX3 ↓	Inhibits PTX3 pathway	Promotes cardiac I/R injury	Cardiac I/R injury	[62]
miR-9 ↑	GOT1 ↓	Inhibits GOT1 pathway	Inhibits melanoma	Melanoma	[45]
miR-182-5p ↑	GPX4 ↓	Inhibits GPX4 pathway	Inhibits I/R-induced kidney injury	I/R-induced kidney injury	[42]
miR-378a-3p ↑	SLC7A11 ↓	Inhibits SLC7A11 pathway	Inhibits I/R-induced kidney injury	I/R-induced kidney injury	[42]
lncRNA-ZFAS1 ↑	miR-150-5p ↓	Inhibits miR-150-5p/CCND2	Promotes DbCM	DbCM	[76]
lncRNA-KCNQ1OT1 ↑	miR-7-5p ↓	Inhibits KCNQ1OT1/miR-7-5p	Promotes ferroptosis	Cardiomyocyte ferroptosis	[77]
lncRNA-XXYLT1-AS2 ↑	AKT ↑ and NF-*κ*B ↑	Activates the AKT-NF-*κ*B signaling pathway	Against the inflammatory response	Atherosclerosis	[71]
lncRNA-UCA1 ↑	miR-873-5p ↓	Inhibits miR-873-5p/XIAP axis	Cardiac protective effect	Myocardial infarction	[72]
lncRNA-LINC00336 ↑	ELAVL1 ↑	Increase the level of CBS	Inhibits ferroptosis	Lung cancer	[73]
lncRNA PVT1 ↑	miR-214 ↓	Inhibits miR-214/TFR1 and p53	Promotes infarct size and ferroptosis	Acute ischemic stroke	[74]
circSnx12 ↑	miR-224-5p ↓	Activates FTH1	Promotes ferroptosis	Heart failure	[84]
lncRNA-p21↓	MDM2 ↑	Inhibits the formation of the p300-p53 complex	Promotes the coronary heart disease	Coronary heart disease	[69]
miR-190a-5p ↓	GLS2 ↑	Activates GLS2 pathway	Protection of myocardial I/R injury	Myocardial I/R injury	[57]
miR-143-3p ↓	GOT1 ↑	Activates GOT1 activity	Inhibits viability of cardiomyocytes	Atrial fibrillation	[60]
miR-30d ↓	ATG5 ↓	Inhibits ATG5 pathway	Promotes the myocardial I/R injury	Myocardial I/R injury	[61]
miR-351 ↓	MLK3 ↑	Activates N JNK/p53 pathway	Promotes myocardial fibrosis	Heart failure	[63]
miRNA-128 ↓	p38*α* ↑	Activates p38a/M-CSF inflammatory signaling pathway	Promotes chronic constipation	Chronic constipation	[85]
circRNA1615 ↓	miRNA152-3p ↓	Inhibits miRNA152-3p/LRP6	Prevents myocardial infarction	Myocardial infarction	[83]

A20: also known as TNF-*α*-induced protein 3; I/R injury: ischemia/reperfusion injury; GPX4: glutathione peroxidase 4; PTX3: pentraxin 3. SLC7A11: solute carrier family 7 member 11; MDM2: mouse double minute 2; DbCM: diabetic cardiomyopathy; MIAT: myocardial infarction associated transcript; MDM2: mouse double minute 2; XXYLT1-AS2: a novel long noncoding RNA; ELAVL1: ELAV-like RNA-binding protein 1; CCND2: cyclin D2; XIAP: X-linked inhibitor of apoptosis protein; GLS2: glutaminase 2; GOT1: glutamic-oxaloacetic transaminase 1; ATG5: autophagy-related 5; MLK3: mixed lineage kinase 3.

**Table 2:** Mechanism of drugs treating CVD.

Diseases	Drugs	Mechanism	Reference
Arteriosclerosis	Erastin	Modulates miR-17–92/A20/ACSL4 axes	[85]
Hypertension	ACEI	Inhibits miR-155-5p to suppressing ACE expression	[86]
Myocardial damage	Simvastatin	Inhibits miR-15a-5p to increase Bcl-2 expression and decreases Bak expression	[87]
Myocardial infarction	Icariside II	Upregulates miR-7-5p to suppress BTG2 expression	[89]
I/R injury	Curcumin	Upregulates miR7-5p and downregulates RelA p65 expression	[88]

ACEI: angiotensin-converting enzyme inhibitor; ACE: angiotensin-converting enzyme; BTG2: BTG antiproliferation factor.
